# Palisaded Granulomatous Dermatitis Associated with Ulcerative Colitis: A Comprehensive Literature Review

**DOI:** 10.7759/cureus.958

**Published:** 2017-01-06

**Authors:** Katherine M Stiff, Philip R Cohen

**Affiliations:** 1 Student, Northeast Ohio Medical University; 2 Department of Dermatology, University of California, San DIego

**Keywords:** palisaded, granulomatous, dermatitis, ulcerative colitis

## Abstract

Palisaded granulomatous dermatitis is an uncommon pathologic condition potentially associated with several disorders. These include drugs, inflammatory bowel disease, multiple myelomas, rheumatoid arthritis, and systemic lupus erythematosus. An illustrative case of a man with palisaded granulomatous dermatitis who subsequently developed ulcerative colitis is described, and the characteristics of other individuals with ulcerative colitis-associated palisaded granulomatous dermatitis are reviewed. PubMed was used to search the following terms: palisaded, interstitial, granulomatous, dermatitis, ulcerative colitis, and neutrophilic. Papers were obtained and references were reviewed. Ulcerative colitis-associated palisaded granulomatous dermatitis is uncommon. Palisaded granulomatous dermatitis-associated ulcerative colitis has been reported in four individuals. The palisaded granulomatous dermatitis appeared from six years prior to diagnosis to 19 years following diagnosis of the patient’s gastrointestinal disease. In addition to individual and grouped papular lesions on the elbows, the morphology of palisaded granulomatous dermatitis can also present as indurated linear plaques overlying the metacarpophalangeal (MCP) joints and proximal fingers.

## Introduction and background

Palisaded granulomatous dermatitis is an uncommon dermatologic condition [1].  The clinical changes most commonly involve symmetric papules, nodules, and plaques on the extremities [1]. The lesions have been described as a “burning rope sign” when they occur as linear cords on the flank [2]. The pathologic changes correspond to skin lesions that may be observed in patients with autoimmune disorders, hematologic malignancies, inflammatory bowel disease, or medications (Table 1) [1-19]. In addition to systemic diseases, palisaded granulomatous dermatitis has also been associated with soy products [1]. An illustrative case of palisaded granulomatous dermatitis in a man whose skin lesions preceded the diagnosis of ulcerative colitis is described and the features of other individuals with ulcerative colitis-associated palisaded granulomatous dermatitis are reviewed. 

**Table 1:** Medications and Conditions Associated with Palisaded Granulomatous Dermatitis

Medications and conditions associated with palisaded granulomatous dermatitis [1-19]	
Autoimmune Disorders	Connective tissue disorders [1]
	Dermatomyositis [3]
	Hepatitis (autoimmune) [4-5]
	Rheumatoid arthritis [6]
	Systemic lupus erythematosus [1-2]
	Systemic sclerosis [7]
Cancer	Hematologic Malignancies:
	Acute promyelocytic leukemia [8]
	Leukemia [9]
	Lymphoma [9]
	Myelodysplastic syndrome [9]
	Paraproteinemia [9]
	Solid Tumors:
	Nasopharyngeal carcinoma [3]
Gastrointestinal Disease	Celiac disease [10]
	Inflammatory Bowel Disease:
	Crohn’s disease [11]
	Ulcerative colitis [12-14]
Medications	Angiotensin converting enzyme inhibitors [15]
	Diuretics [15]
	Tumor necrosis factor alpha inhibitors [16]
Other	Antiphospholipid syndrome [1, 17]
	Behcet's disease [18]
	Diabetes mellitus (Type 1) [10]
	Sarcoidosis [19]
	Systemic vasculitis [19]

### Illustrative case

A 45-year-old man presented for evaluation of skin lesions on his elbows and hands. The lesions had been present for 12 years and were asymptomatic. His past medical history was significant for ulcerative colitis, diagnosed six years prior to his visit. His inflammatory bowel disease had been treated with several agents; he experienced improvement of the skin lesions when flares of his ulcerative colitis were treated with systemic corticosteroids.

Cutaneous examination showed individual and confluent dermal papules ranging in size from 2-4 mm on his elbows (Figure 1). His dorsal hands showed prominent dermal nodules overlying the metacarpophalangeal (MCP) joints of the second, third, and fourth digits on his right hand and the third, fourth, and fifth digits on his left hand (Figure 2). In addition, on the third digit of his right hand and the fourth digit of his left hand, a linear plaque with a rope-like appearance extended from the MCP joint towards the proximal interphalangeal (PIP) joint (Figure 2). When his hands were fisted, the lesions blanched and were accentuated (Figure 3).

**Figure 1:** Right elbow lesions of palisaded granulomatous dermatitis Distant (a) and closer (b and c) views of the right elbow show individual and confluent erythematous papules. Some of the papules are arranged in an annular distribution.

**Figure 2:** Palisaded granulomatous dermatitis involving the hands Distant (a) and closer (b and c) views of both hands; the right hand (b) and the left hand (c) show nodules overlying the second, third, and fourth metacarpophalangeal (MCP) joints of the right hand and the third, fourth, and fifth MCP joints of the left hand. In addition, the right hand (b) and the left hand (c) show linear plaques extending from the third (right hand) and fourth (left hand) MCP joint towards the proximal interphalangeal (PIP) joint which were morphologically cord-like or rope-like.

**Figure 3:** Palisaded granulomatous dermatitis lesions blanch when hands are fisted The lesions are blanched and accentuated when the right (a) and left (b) hand is fisted.

Microscopic examination of biopsies from both the right elbow (Figure 4) and right hand (Figure 5) showed similar pathologic changes. Palisading granulomas consisting predominantly of lymphocytes and histiocytes were present throughout the dermis. Occasional neutrophils were also noted in the granulomatous inflammation (Figures 4a, 4b, 5a, 5b). There was degeneration of the collagen in the center of granulomas with periodic acid-Schiff (PAS) positive staining material, consistent with fibrin deposition (Figures 4c, 4d, 5c, 5d). Mucin was present throughout the dermis and was not increased within the central area surrounded by the granulomas (Figures 4e, 4f, 5e, 5f).

**Figure 4:** Histology of lesion on the right elbow Microscopic examination of a skin lesion on the right elbow shows palisaded granulomas that extend into the mid-reticular dermis (a and b). Closer examination (b) shows histiocytes and lymphocytes palisading around area of degenerated collagen. Fibrin deposition is noted in the center of the granulomas (c and d). Mucin is present throughout the dermis; however, it is not increased within the altered collagen surrounded by the granuloma (e and f). (hematoxylin and eosin: x2 = a, x20 = b; periodic acid-Schiff: x4 = c, x40 = d; colloidal iron: x4 = e, x20 = f)

**Figure 5:** Histology of lesion on right third metacarpophalangeal joint Microscopic examination of a biopsy from the skin lesion located on the right third metacarpophalangeal joint shows similar pathologic changes to those on the elbow. The granulomatous inflammation extends into the deep reticular dermis (a and b). Fibrin is noted to be present (c and d) and mucin is noted to be absent within the altered dermal collagen surrounded by the granuloma (e and f). (hematoxylin and eosin: x2 = a, x20 = b; periodic acid-Schiff: x4 = c, x40 = d; colloidal iron: x10 = e, x40 = f)

Correlation of the clinical presentation and pathologic changes established a diagnosis of palisaded granulomatous dermatitis. The patient’s history of ulcerative colitis suggests that the dermatitis was associated with his inflammatory bowel disease. Clobetasol propionate 0.05% cream was prescribed twice daily to be applied to the lesions. The patient did not return for follow-up. 

## Review

### Palisaded granulomatous dermatitis

History

Palisaded granulomatous dermatitis is an uncommon condition associated with characteristic clinical and pathological features. It was originally described under the nomenclature “allergic granulomatosis” by Churg and Strauss in 1951 [20]. Subsequently, it was renamed “palisaded neutrophilic and granulomatous dermatitis” by Chu, et al. in 1994 [21]. This condition appears under several other nomenclatures in literature: Churg-Strauss granuloma [22], cutaneous extravascular necrotizing granuloma [22], interstitial granulomatous dermatitis with arthritis [23], linear subcutaneous bands [24], and rheumatoid papules [25].

Clinical Presentation

The lesions generally appear as symmetric erythematous to flesh-colored papules on the extensor surfaces of the upper extremities, particularly on the elbows [7]. Individual lesions may coalesce into plaques or annular rings. The lesions vary from asymptomatic to tender and painful.

In some patients, the dermatitis is characterized by linear, indurated, erythematous lesions with a cord appearance. These lesions are referred to as having a “rope sign” [2]. One patient not only had typical papules on his elbows but also had linear, indurated lesions on his right and left dorsal hands (Figure 2). To the best of our knowledge, this is an uncommon presentation of the rope sign.

Pathology

There are a variety of pathologic changes associated with palisaded granulomatous dermatitis. The descriptive designation of the condition in individual patients often reflects the predominant cellular inflammatory infiltrate of the granulomas. The histologic appearance ranges from lymphocytes or histiocytes or eosinophils, and/or sparse neutrophils [26] to dense neutrophilic infiltrates with degenerated collagen and palisading granulomas with fibrosis and neutrophilic debris [21]. In one patient, granulomas were present in the dermis with degeneration of collagen in the central areas. Fibrin was present in the granulomas, and mucin was not prominent.

Clinical Differential Diagnosis

The clinical differential diagnosis is varied. It includes granuloma annulare, interstitial granulomatous dermatitis, leukocytoclastic vasculitis, and urticaria (Table 2) [6, 19, 27-28]. Pathologic features enable the conditions to be differentiated. For example, mucin is more prominent in the central area of the granuloma in granuloma annulare and is less common or absent in palisaded granulomatous dermatitis. It remains to be established whether interstitial granulomatous dermatitis should be included under the broader category of palisaded neutrophilic granulomatous dermatitis due to the overlapping clinical and histologic features between these two disorders [1].

Pathologic Differential Diagnosis

The pathologic differential diagnosis includes rheumatoid nodules. These are usually deeper in the dermis and have more sclerosis in the area surrounded by the granuloma. It also includes neutrophilic dermatoses, such as bowel-associated dermatosis-arthritis syndrome, erythema elevation diutinum, leukocytoclastic vasculitis, pyoderma gangrenosum, and Sweet’s syndrome (Table 2) [6, 19, 27-28].

**Table 2:** Differential Diagnosis of Palisaded Granulomatous Dermatitis

Clinical differential diagnosis [6, 19]	Pathologic differential diagnosis [27-28]
Erythema Elevatum Diutinum	Abscess/cellulitis
Granuloma annulare	Bowel (intestinal) bypass syndrome
Interstitial granulomatous dermatitis	Bowel associated dermatosis-arthritis syndrome
Leukocytoclastic vasculitis	Erythema elevatum diutinum
Sarcoidosis	Granuloma faciale
Urticaria	Halogenoderma
	Leukocytoclastic vasculitis
	Neutrophilic urticarial dermatosis
	Pyoderma gangrenosum
	Rheumatoid nodules

Pathogenesis

The pathogenesis of palisaded granulomatous dermatitis remains to be established. Palisaded granulomatous dermatitis may occur as an idiopathic disorder; however, it is often associated with other conditions or medications (Table 1) [1-19].  Ulcerative colitis-associated palisaded granulomatous dermatitis is rare. To the best of our knowledge, including our patient, it has only been described in four individuals (Table 3) [12-14].

**Table 3:** Cases with Ulcerative Colitis-Associated Palisaded Granulomatous Dermatitis Abbreviations: C = case, Col = colchichine, CP = clobetasol proprionate cream, CR = current report, Cs = corticosteroid, DM = dapsone monotherapy, G = gender, GD = granulomatous dermatitis, KI = potassium iodine, L = left, M = men, MCP = metacarpophalangeal, Mino = minocycline, NIGD = non-interstitial granulomatous dermatitis, NSAIDS = non-steroidal anti-inflammatory drugs, PGD = palisaded granulomatous dermatitis, PIP = proximal interphalangeal, PNGD = palisaded neutrophilic granulomatous dermatitis, Pred = prednisone, R = right, UC = ulcerative colitis, W = women, y = year ^a^ Ulcerative colitis preceded (p) diagnosis of palisaded granulomatous dermatitis or follows (f) diagnosis of palisaded granulomatous dermatitis by the stated number of years. ^b^ The patient had taken oral NSAIDs for seven months and topical application of the strongest class of Cs ointment for two weeks with no success. She was then started on oral KI at 900 mg/day; however, this was ineffective and discontinued after two weeks. Subsequently, oral DDS was started at 75 mg/day, and symptoms were gone after six months. ^c ^The onset of palisaded granulomatous dermatitis occurred after the patient’s colectomy. ^d ^The patient was treated with pred at 50 mg and improved within 36 hours. She remained free of lesions during the pred taper over 10 days. However, she had recurrence of induration and erythema of right forearm on the last day of pred 10 mg; therefore, she was started on 50 mg pred along with mino 100 mg twice daily. After three days of no improvement, col 0.6 mg twice daily was added. ^e ^The patient did not return for follow-up.

C	G	Age (y)	UC p/f^a^	Site	Morphology	Path	Tx	Ref
1	W	22	p2	L chest	Painful erythematous plaque	GD	Resolved after colonic resection	12
2	W	32	p19	Hands, MCP and PIP joints, L big toe	Tender papules, nodules, and erythematous plaques	PNGD	NSAIDs, Cs ointment, KI, DM^b^	13
3	W	68	p^c^	R arm, L elbow	Indurated, erythematous, tender plaque (R arm), Shiny violaceous, non-tender plaque (L arm)	NIGD	Pred, Mino, Col^d^	14
4	M	45	f6	Elbows, Hands, MCP and PIP joints	Asymptomatic individual and grouped papules (elbows), nodules (hands), and indurated linear plaques (hands)	PGD	CP 0.05%^e^	CR

### Ulcerative colitis

Epidemiology

Ulcerative colitis is the most common form of inflammatory bowel disease. It is a mucosal disease with an incidence of 1.2 to 20.3 cases per 100,000 persons per year, and a prevalence of 7.6 to 246.0 cases per 100,000 per year. Inflammatory bowel disease is linked to smoking, high fat and sugar diets, medications, stress, and high socioeconomic status [25].

Pathogenesis

The pathogenesis of inflammatory bowel disease may be a lack of tolerance to the microorganisms in the gut. It is characterized by a TH2 predominance. When present, it is always in the colon and rectum [25].

Clinical Presentation and Pathology

The characteristic feature of ulcerative colitis is bloody diarrhea with or without mucus. It has a gradual onset with spontaneous remission and relapses. The histologic features show inflammation limited to the mucosal layer and infiltrates of lymphocytes, plasma cells, and granulocytes. In addition to palisaded granulomatous dermatitis, cutaneous manifestations of ulcerative colitis include cutaneous polyarteritis nodosa, erythema nodosum, necrotizing vasculitis, oral aphthous ulcers, pyoderma gangrenosum, pyostomatitis vegetans, Sweet’s syndrome, and thrombosis [24-25].

Treatment

The first line treatment of ulcerative colitis includes sulfasalazine and 5-aminosalicylates. If the first line treatment is unsuccessful, glucocorticoids may be used. A colectomy can be curative in patients with ulcerative colitis but is a treatment of last resort [25].

### Ulcerative colitis-associated palisaded granulomatous dermatitis

Epidemiology

Ulcerative colitis-associated palisaded granulomatous dermatitis has occurred in three women (ranging in age from 22 to 68 years at the time of diagnosis of the skin condition, median = 32) and one man, whose skin lesion appeared when he was 33 years old (Table 3) [12-14].

Clinical Presentation

The lesions in three of the patients were tender; they were asymptomatic in one patient. One woman had a lesion on her left elbow that was asymptomatic, in addition to a tender lesion of the right arm. Skin lesions were present on the dorsal hands (two patients), elbow (two patients), and chest (one patient). One patient also had an indurated papule on her left big toe, in addition to the lesions on her hands (Table 3) [12-14].

The morphology of the palisaded granulomatous dermatitis lesions was papules or plaques that were individual or coalesced. None of these patients had linear indurated lesions on their flanks. However, one patient not only had nodular lesions on his MCP joints but also a cord-like linear lesion on his dorsal right and left hands extending from the MCP joint distal towards the PIP joint.

Pathology

Microscopic examination of the lesions in the individuals with ulcerative colitis all showed similar features: granulomas in the dermis. Two of the patients had dense neutrophilic infiltrate in the granulomas (Cases 1 and 2). The other two patients had a predominantly lymphohistiocytic infiltrate with occasional neutrophils (Cases 3 and 4).

Temporal Association of Palisaded Granulomatous Dermatitis and Ulcerative Colitis

The onset of granulomatous dermatitis with regards to the diagnosis of ulcerative colitis varied. The skin condition presented as early as six years prior to diagnosis to as late as 19 years following the diagnosis. One patient also had myelodysplastic syndrome and developed the skin condition post-colectomy. Hence, her dermatitis may have been associated with the myelodysplastic syndrome.

Treatment

Management of palisaded granulomatous dermatitis in patients with ulcerative colitis has included oral colchicine, dapsone, minocycline, and/or prednisone; topical corticosteroids have also been utilized as a therapy. One patient noted improvement of his lesions when he was treated with systemic corticosteroids for an ulcerative colitis flare. Treatment with a high-potency topical corticosteroid was initiated; however, the patient was not able to be evaluated at follow-up. Other patients were successfully treated with either dapsone monotherapy, prednisone with minocycline, or colchicine. One patient’s skin condition resolved after a partial colectomy (Table 3) [12-14].

Other patients with granulomatous dermatitis not associated with ulcerative colitis have been successfully treated with cyclosporine, dapsone, hydroxychloroquine, methotrexate, and prednisone. Dapsone has demonstrated a greater treatment success compared to other oral therapies [25, 30].

## Conclusions

Palisaded granulomatous dermatitis is an uncommon cutaneous condition that is typically associated with an underlying disorder or a systemic medication. Ulcerative colitis-associated palisaded granulomatous dermatitis has only been described in four individuals, including the patient in our report. Ulcerative colitis patients have developed the skin lesions as early as six years prior to diagnosis to as late as 19 years after the onset of their inflammatory bowel disease. Similar to palisaded granulomatous dermatitis patients without ulcerative colitis, papules on the elbows is the most common presentation in ulcerative colitis-associated palisaded granulomatous dermatitis. Although none of the ulcerative colitis patients had classic-appearing rope-like lesions on their flanks, one patient did have a cord-like appearance of his lesions on the right and left dorsal hands extending from his MCP joint towards his PIP joint. The skin lesions of palisaded granulomatous dermatitis in patients with ulcerative colitis responded to dapsone and corticosteroids, similar to lesions of palisaded granulomatous dermatitis in patients without ulcerative colitis. 
